The article "Effect of Transumbilical Single-Port Laparoscopic-Assisted Duhamel Operation on Serum CRP and IL-6 Levels in Children with Hirschsprung's Disease" was retracted in 2023. Reasons: signs of a paper mill; suspected computer-generated content; unreliable results or conclusions; lack of ethics approval or compliance.

# Effect of Transumbilical Single-Port Laparoscopic-Assisted Duhamel Operation on Serum CRP and IL-6 Levels in Children with Hirschsprung's Disease

**DOI:** 10.1155/2022/8349851

**Published:** 2022-03-02

**Authors:** Miao Wang, Wenshuai Pang, Lixia Zhou, Jiansu Ma, Shasha Xie

**Affiliations:** Xingtai People's Hospital, Hebei, Xingtai 054000, China

## Abstract

**Objective:**

To explore the clinical intervention effect of transumbilical single-port laparoscopic-assisted Duhamel operation on children with Hirschsprung's disease (HD) and to analyze the effect of treatment on children with serum C-reactive protein (CRP) and interleukin-6 (IL-6) effects.

**Methods:**

Retrospectively select 80 children with HD who underwent surgery in our hospital from May 2017 to May 2020 as the research subjects and they are classified as group A according to the difference of the children's surgical procedures (receiving transumbilical single-port laparoscopic-assisted Duhamel surgery, 40 cases) and group B (receiving conventional laparoscopic surgery, 40 cases), compare the perioperative period (operating time, intraoperative blood loss, surgical posthospitalization, and postoperative gastrointestinal function recovery time), early postoperative complications (perianal dermatitis, urinary retention, enterocolitis, and anastomotic leakage), and late postoperative complications (anastomotic stenosis, dirty stool, recurrence of constipation, and enterocolitis), compare the differences in the levels of CRP and IL-6 between the two groups of children before and after the operation, and conduct a 1-year follow-up of the two groups of children to compare the long-term defecation status.

**Results:**

The surgical time of children in group A, postoperative hospitalization time, and postoperative gastrointestinal function recovery time were significantly shorter than those of group B, and the differences between groups were statistically significant (*P* < 0.05). A group of patients: the total incidence of postearly complications was 5.00% lower than 22.50% (*P* < 0.05) in group B (*P* < 0.05), and the total incidence of previous complications after group A of patients was 10.00% lower than 27.50% of group B (*P* < 0.05). The two groups of serum CRP and IL-6 in two groups were not statistically significant (*P* > 0.05), and the serum CRP and IL-6 levels of children in group A after surgery were 3 days. It is obviously lower than those in group B, and the differences between groups have statistical significance (*P* < 0.05). At 1 month after surgery, the average bowel movement time in group A is significantly lower than those of group B (*P* < 0.05); during the 1–12 months, the difference between the defecation frequency group of the group A and group B did not have statistically significance (*P* > 0.05).

**Conclusion:**

Transumbilical single-port laparoscopic assistant Duhamel operation of HD has a good intervention effect, compared to traditional laparoscopic surgery, the operation time, postoperative hospitalization time, and postoperative gastrointestinal function recovery time, and also help to reduce postoperative near-long complications The incidence improves the stress reactions and long-term defecation functions in children.

## 1. Introduction

Hirschsprung's disease (HD) is one of the common types of pediatric digestive tract developmental deformities [1]. Its incidence ranks second among congenital malformations of the digestive system. The lesions in children are characterized by the intermuscular nerves at the end of the intestine. The lack of plexus and submucosal ganglion cells causes the intestinal tube to be in a state of spasm, loses normal peristaltic function, and makes the intestine in a narrow state [2, 3]. The clinical manifestations of children with HD are mainly refractory constipation, abdominal distension, malnutrition, and stunted growth or Hirschsprung's disease with enterocolitis. In recent years, the improvement of diagnosis and treatment technology has enabled 70–90% of cases to be diagnosed in the neonatal period, and only a few children with milder clinical symptoms are not diagnosed until adolescence or adulthood [4, 5]. Since the long-term development of this disease will cause the expansion of the proximal colon to continue to increase, the patient's constipation symptoms will continue to increase or even develop into acute intestinal obstruction, and it is recommended to carry out early active surgical treatment for such children [6].

The current surgical treatment principle of HD is to remove the intestinal segment without ganglion cells and the expanded intestinal segment [7]. Since the Swenson procedure was applied to the clinical treatment of HD in 1948, various modified procedures such as by Duhamel, Rehbein, and Sovae have continued emerging, providing medical workers with a variety of options [8]. Since the 1980s, minimally invasive techniques represented by laparoscopy have been gradually used in the radical resection of HD. In 1999, laparoscopic-assisted Soave endorectal evacuation was recognized as the gold standard for HD treatment. With the continuous improvement of laparoscopic technology and the continuous improvement of surgical instruments, scarless surgery such as single incision through the umbilical or through the natural cavity has become the mainstream treatment for HD [9, 10]. This study is currently planning to take 80 children with HD admitted to our hospital from May 2019 to May 2020 as the research object.

A comparative analysis by means of statistical measures between transumbilical single-port laparoscopic-assisted Duhamel surgery and conventional laparoscopic surgery is carried out. The pros and cons of the surgical treatment of children with HD are compared in order to provide more detailed theoretical support for improving the prognosis of children with HD.

## 2. Materials and Methods

### 2.1. General Information

We retrospectively selected 80 children with HD who underwent surgery in our hospital from May 2017 to May 2020 as the research objects and divided them into group A according to the difference of the children's surgical procedures (receiving transumbilical single-port laparoscopic-assisted Duhamel surgical treatment, 40 cases) and group B (receiving conventional laparoscopic surgery, 40 cases). The two groups of gender, age, weight, and lesion are included, and the intergroup differential comparisons were implemented. As a result, the difference between the above data groups in the two groups did not have statistically significant (*P* > 0.05), suggesting comparable (Table 1).

Inclusion criteria: those who have been diagnosed with Hirschsprung's disease, those who are ineffective in conservative treatment and have indications for surgery, and the case data are complete.

Exclusion criteria: patients with congenital malformations or organic diseases, combined with severe heart, liver, and kidney function failures, combined with malignant tumor, patients with hematological diseases, included other unfinished clinical researchers.

### 2.2. Intervention Methods

Children in group A underwent transumbilical single-port laparoscopic-assisted Duhamel operation, received conventional antibiotic treatment before operation, and selected general anesthesia for tracheal intubation. A longitudinal incision was made at the umbilical fossa of the children, and a trocar was placed to create an artificial pneumoperitoneum environment (8–12 mmHg); the child's lithotomy position was used to dilate the anus, and the rectal mucosa was incised obliquely at a distance of 1 cm from the dentinal line and 2 cm from the anterior wall of the rectal mucosa. Mesocolon, pull the free colon to the right lower abdomen, push the small intestine to the left upper abdomen, straighten out the mesenteric blood vessels, transfer the operation to the perineum, cut off the rectal muscle sheath through the anus, and drag the free colon out of the body and cut it off. And finally, implement the colorectal anastomosis. The preoperative operation of the children in group B was the same as that in group A. The same incision was made in the umbilical area, and a laparoscope with a 5 mm operating channel was inserted. After the situation was verified, a 5 mm trocar was placed in the left and right lower abdomen, and an ultrasonic knife edge was used. Dissociate around the pelvic cavity and rectum and process the colonic mesangium and blood vessels until the normal intestinal canal. After dissociation is completed, perform perineal operations and finally suture the edge of the colon and rectal mucosa.

### 2.3. Observation Indicators and Evaluation Standards

General surgical indicators of the two groups of children, including operation time, postoperative hospitalization time, intraoperative blood, and postoperative gastrointestinal function recovery time; early postoperative complications of the two groups of children include perianal dermatitis, incidence rates of urinary retention, enterocolitis, and secondary operations; the incidence of long-term postoperative complications of the two groups of children including anastomotic stenosis, feces, constipation recurrence, and enterocolitis; serum CRP and IL-6 levels of the two groups of children when they were admitted to the hospital and 3 days after the operation; the defecation function evaluation of the two groups of children after 12 months of follow-up.

### 2.4. Statistical Methods

The collected data are entered into the Excel form, statistical SPSS 22.0 software was used for data analysis, and a normal distribution test on the collected data was carried out, such as data compliance with normal distribution, counting data is indicated by (*n* (%)), differential analysis selection card foundation inspection, metrology data representation (measurement) difference analysis, and *t-*test was selected. Take *P* < 0.05 as a statistical significance [11].

## 3. Results

### 3.1. Comparison of Differences in Perioperative Indicators between the Two Groups of Children

In comparison, the operation time of children in group A, postoperative hospitalization time, and postoperative gastrointestinal function recovery time were significantly shorter than those of the group B, and the difference in groups had statistically significance (*P* < 0.05), and the intraoperative blood volume is two. The difference in groups does not have statistical significance (*P* > 0.05) (Figure 1).

The comparison showed that the operation time, postoperative hospital stay, and postoperative gastrointestinal function recovery time of group A were significantly shorter than those of group B. The differences between groups are statistically significant. It is of statistical significance (*P* < 0.05); the difference between the two groups in the intraoperative blood loss did not have statistically significance (*P* > 0.05). It means that the difference between the same index group is statistically significant.

### 3.2. Comparison of the Incidence of Early Postoperative Complications in the Two Groups

Statistics showed that 1 case of perianal dermatitis and 1 case of enterocolitis occurred in group A. The total incidence of complications was 5.00%. In group B, there were 3 cases of perianal dermatitis, 1 case of urinary retention, and 5 cases of enterocolitis. The total incidence rate was 22.50%, and the difference between the individual complications of the individual complications was not statistically significant (*P* > 0.05), and the total incidence of complications was lower than that in group B (*P* < 0.05) (Table 2, Figure 2).

There was no statistically significant difference in the two groups in recent complications after surgery. The total incidence of recent complications in groups was significantly lower than those in group B (*P* < 0.05). The comparison between the same indicator group is statistically significant.

### 3.3. Comparison of the Incidence of Long-Term Complications after the Operation of the Two Groups of Children

Statistics showed that 2 children in group A had postoperative fecal contamination, 2 cases of enterocolitis, and the total complication rate was 10.00%. In group B children, postoperative anastomotic stenosis occurred in 1 case, fecal contamination was in 5 cases, constipation recurred in 1 case, and 4 cases of enterocolitis; the total incidence of complications was 27.50%. The total incidence of comparative complications in group A was lower than those in group B (*P* < 0.05) (Table 3, Figure 3).

Compared with 2 cases of fecal infection and 2 cases of enterocolitis in group A, the total incidence of postoperative complications in group B was 10.00%. The incidence of anastomotic stoma was in group B, including 1 case of stenosis, 5 cases of fecal contamination, 1 case of constipation, and 4 cases of enterocolitis. The total incidence of complications was 27.50%. It can be concluded that the incidence of complications in group A is lower than that in group B (*P* < 0.05). This means that the difference between the same finger array is statistically significant.

### 3.4. Differences in Serum CRP and IL-6 Levels between the Two Groups before and after Operation

At the time of admission, the two groups of children were collected in the empty stomach of the two groups, and preoperative and postoperative serum CRP and IL-6 levels were detected after surgery. Differential differences between the sexy fraternal CRP and IL-6 were not statistically significant (*P* > 0.05), and serum CRP and IL-6 levels in group A were significantly lower than those in group B, and the difference in groups was significantly lower than those in the group. It has statistically significance (*P* < 0.05), while serum CRP and IL-6 levels in two groups of children before surgery were significantly reduced (*P* < 0.05) (Table 4, Figure 4).

### 3.5. Differences in Long-Term Prognosis Assessment between the Two Groups

Assess the long-term prognosis of the two groups. The results show that at 1 month after surgery and 3 months follow-up, the average bowel movement of the A group is significantly lower than that of group B (*P* < 0.05); 6 months after surgery, 9 months after surgery, and 12 months after surgery, the difference in the defecation time group of group A and group B did not have statistically significance (*P* > 0.05). The difference between the two groups of patients during 1–12 months after surgery did not have statistically significance (*P* > 0.05) (Figures 5 and 6).

As shown in Figure 6, for 12 months, during 1–12 months after surgery, the difference in the defecation frequency group in group A and group B did not have a statistical significance (*P* > 0.05).

## 4. Discussion

Hirschsprung's disease (HD) was first formally named in 1894. At first, medical workers believed that the pathological feature of the disease was expansion of the colon and the formation of Hirschsprung's disease led to constipation [12]. It was not until 1948 that Swenson discovered that the pathological feature of HD was stenosis of the distal bowel through barium enema and finally confirmed that its pathological mechanism was the loss of ganglion cells in the stenosis of the colon, which caused the expansion of the proximal colon [13, 14]. HD is currently a relatively common gastrointestinal malformation in pediatric surgery. The incidence is relatively high in the Middle East worldwide, and the incidence in Europe is relatively low. My country is a high-risk group of HD [15, 16].

This study established a control group to demonstrate in detail the advantages and disadvantages of applying transumbilical single-port laparoscopic-assisted Duhamel surgery and traditional laparoscopic surgery in the surgical treatment of children with HD. The results show that compared with traditional laparoscopic surgery in group B of children, children in group A who underwent transumbilical single-port laparoscopic-assisted Duhamel surgery had obvious advantages in terms of operation time, postoperative hospital stay, and postoperative gastrointestinal function recovery time, which are comparable to the results of other scholars [17]. The results of a comparative study conducted on 109 children with HD showed that compared with traditional laparoscopic surgery, transumbilical laparoscopic surgery has the advantages of less trauma and faster recovery after surgery, which is convenient for shortening the postoperative hospital stay [18]. The author of this article analyzes and believes that transumbilical single-port laparoscopic surgery is a modified operation that can be inserted into the umbilical laparoscopic to explore the lesions and complete the perineal rectal mucosal dissection. On the one hand, this operation only has a hidden incision in the umbilical area. It is easy for parents to accept, and on the other hand, it effectively eliminates the “chopstick effect” brought by the same direction operating equipment, which is convenient for intraoperative operation [19].

The article also analyzes the incidence of short and long-term complications in children undergoing two types of surgery. The results show that group A has obvious advantages in terms of both short-term and long-term complications. The author of this article analyzes and believes that the emergence of complications is an important reason for the poor prognosis of children. In this study, the incidence of short-term and long-term complications after surgery in group A was low. The reason may be related to the following transumbilical single-port laparoscopic-assisted Duhamel surgery advantages: comprehensive exploration of the abdominal cavity during the operation can accurately determine the diseased intestine; it can better preserve the vascular arch of the intestine edge, reduce the damage to the external anal sphincter, avoid excessive traction on the sigmoid colon, and reduce postoperative anastomotic leakage, the emergence of feces, and the rapid recovery of defecation function in children after surgery; the use of NOTES surgical instruments during surgery is avoided, and medical costs are reduced [20, 21]. In fact, this point is also reflected in the levels of serum CRP and IL-6 in the two groups of children after surgery. On the one hand, serum CRP and IL-6 can be used as indicators to reflect the postoperative inflammatory status of the children, and on the other hand, it can also reflect the degree of stress in children during operation [22, 23]. The abovementioned indicators in group A are lower than those in group B after surgery, which indicates that the stress stimulation in group A is lower during operation. The perioperative indexes of children in group A are better than those in group B.

Finally, the article also conducted a preliminary analysis of the long-term prognosis of the two groups of children. The results showed that the average defecation time of the children in group A was lower than that of group B in the early postoperative period, but the defecation function of the two groups of children was not obvious in the long-term. The difference indicates that the two types of surgery have a significant improvement effect on the long-term defecation function of children, but the difference between the groups is not obvious. It is recommended that in terms of reducing the early postoperative stress response and the incidence of complications in children, try to choose transumbilical single-port laparoscopic-assisted Duhamel surgery for children with HD [24].

In summary, transumbilical single-port laparoscopic-assisted Duhamel surgery has a better intervention effect on children with HD. Compared with traditional laparoscopic surgery, it can significantly shorten the operation time, postoperative hospital stay, and postoperative gastrointestinal function recovery time, and it also helps to reduce short and long-term postoperative complications, incidence rate and improve postoperative stress response and long-term bowel function in children.

## Figures and Tables

**Figure 1:** Comparison of perioperative index differences in children in two groups.

**Figure 2:** The incidence of early complications in the two groups.

**Figure 3:** The incidence of postoperative complications after two groups.

**Figure 4:** The serum CRP and IL-6 levels of children in two groups before and after surgery. The serum CRP and IL-6 levels of children in group A were significantly lower than those in group B, and the difference in groups was significantly lower than those of group B, and the difference in groups was statistically significant (*P* < 0.05). ^#^The comparison between the same indicator group is statistically significant.

**Figure 5:** Postoperative defecation time follow-up for two groups of patients. For 12 months at 1 month after surgery, the average bowel movement of the A group was significantly lower than those of group B (*P* < 0.05); 6 months after surgery, 9 months after surgery, and 12 months after surgery, the difference in the blasting time group in groups A and B did not have statistically significance (*P* > 0.05). ^#^The comparison between the same indicator group is statistically significant.

**Figure 6:** After the two groups of patients were followed up.

**Table 1:** Comparison of baseline data differences in two groups ($\bar{x}\pm s$)/(*n* (%)).

Baseline data		Group A (*n* = 40)	Group B (*n* = 40)	*t*/*χ*^2^	*P*
Gender	Male	21	19	0.05	0.823
	Female	20	20		
Average age (years)		2.79 ± 0.22	2.81 ± 0.19	0.435	0.665
Average weight (kg)		15.19 ± 1.22	15.23 ± 1.09	0.155	0.877
Average height (cm)		0.81 ± 0.05	0.79 ± 0.07	1.47	0.146
Type of lesion	Common type	34	35	0.105	0.745
	Long section	6	5		

**Table 2:** Comparison of the incidence of early postoperative complications between the two groups of children (*n* (%)).

Group	Number of cases	Perianal dermatitis	Urinary retention	Enterocolitis	Second surgery	Total incidence
Group A	40	1 (2.50)	0 (0.00)	1 (2.50)	0 (0.00)	2 (5.00)
Group B	40	3 (7.50)	1 (2.50)	5 (12.50)	0 (0.00)	9 (22.50)
*X* ^2^	—	1.053	1.013	2.88	0.0	5.165
*P*	—	0.305	0.314	0.090	1.0	0.023

**Table 3:** Comparison of the incidence of long-term postoperative complications between the two groups of children (*n* (%)).

Group	Number of cases	Anastomotic stenosis	Dung	Recurrence of constipation	Enterocolitis	Total incidence
Group A	40	0 (0.00)	2 (2.50)	0 (0.00)	2 (5.00)	4 (10.00)
Group B	40	1 (2.50)	5 (12.50)	1 (2.50)	4 (10.00)	11 (27.50)
*X* ^2^	—	1.013	1.409	1.013	0.721	4.021
*P*	—	0.314	0.235	0.314	0.396	0.045

**Table 4:** Differences in serum CRP and IL-6 levels between the two groups of children before and after surgery ($\bar{x}\pm s$).

Group	Number of cases	CRP (mg/ml)		IL-6 (pg/ml)	
		On admission	3 d after operation	On admission	3 d after operation
Group A	40	39.29 ± 5.44	15.49 ± 2.11^#^	36.98 ± 2.11	25.67 ± 4.33^#^
Group B	40	39.98 ± 4.98	20.11 ± 1.98^#^	37.32 ± 1.98	29.11 ± 3.98^#^
*t*	—	0.592	10.098	0.743	3.699
*P*	—	0.556	<0.001	0.460	0.000

Compared with admission, ^#^*P* < 0.05.

## Data Availability

The data used to support the findings of this study are available from the corresponding author upon request.
